The article "ADVIAN: Alzheimer's Disease VGG-Inspired Attention Network Based on Convolutional Block Attention Module and Multiple Way Data Augmentation" was retracted in 2023. Reasons: compromised peer review; unreliable results or conclusions.

# ADVIAN: Alzheimer's Disease VGG-Inspired Attention Network Based on Convolutional Block Attention Module and Multiple Way Data Augmentation

**DOI:** 10.3389/fnagi.2021.687456

**Published:** 2021-06-18

**Authors:** Shui-Hua Wang, Qinghua Zhou, Ming Yang, Yu-Dong Zhang

**Affiliations:** ^1^Key Laboratory of Child Development and Learning Science (Southeast University), Ministry of Education, Nanjing, China; ^2^School of Mathematics and Actuarial Science, University of Leicester, Leicester, United Kingdom; ^3^School of Informatics, University of Leicester, Leicester, United Kingdom; ^4^Department of Radiology, Children's Hospital of Nanjing Medical University, Nanjing, China

**Keywords:** Alzheimer‘s disease, convolutional block attention module, VGG, transfer learning, deep learning, attention network, data augmentation

## Abstract

**Aim:** Alzheimer's disease is a neurodegenerative disease that causes 60–70% of all cases of dementia. This study is to provide a novel method that can identify AD more accurately.

**Methods:** We first propose a VGG-inspired network (VIN) as the backbone network and investigate the use of attention mechanisms. We proposed an Alzheimer's Disease VGG-Inspired Attention Network (ADVIAN), where we integrate convolutional block attention modules on a VIN backbone. Also, 18-way data augmentation is proposed to avoid overfitting. Ten runs of 10-fold cross-validation are carried out to report the unbiased performance.

**Results:** The sensitivity and specificity reach 97.65 ± 1.36 and 97.86 ± 1.55, respectively. Its precision and accuracy are 97.87 ± 1.53 and 97.76 ± 1.13, respectively. The F1 score, MCC, and FMI are obtained as 97.75 ± 1.13, 95.53 ± 2.27, and 97.76 ± 1.13, respectively. The AUC is 0.9852.

**Conclusion:** The proposed ADVIAN gives better results than 11 state-of-the-art methods. Besides, experimental results demonstrate the effectiveness of 18-way data augmentation.

## Background

Alzheimer's disease (AD) is a neurodegenerative disease, which affects 60%−70% of all cases of dementia (Alhazzani et al., 2020). The main symptom of AD is difficulty in short-term memory. As AD progressively worsens, patients exhibit symptoms such as mood and cognition (Lee et al., 2019), motivation loss, speech and language problems (Petti et al., 2020), spatial disorientation (Puthusseryppady et al., 2020), sleep behaviors (Mather et al., 2021), etc. These symptoms lead to a significant decline in quality of life and an increase in care-taker burden (Scheltens et al., 2016; Fulton et al., 2019). AD's etiology is damage to brain cells observable on imaging scans (Fulton et al., 2019) as the atrophy of anatomical structures like the cerebral cortex. The atrophy is caused by amyloid plaque (Ferreira et al., 2021) formation and neurofibrillary tangles (Kumari and Deshmukh, 2021). Manual differential diagnosis of AD is lab-intense, onerous, and expensive due to various mental and physical tests, laboratory and neurological tests, and neuroimaging scans (Senova et al., 2021) [computed tomography (CT), positron emission tomography (PET), or magnetic resonance imaging (MRI)] which requires professional experts.

The article "ADVIAN: Alzheimer's Disease VGG-Inspired Attention Network Based on Convolutional Block Attention Module and Multiple Way Data Augmentation" was retracted in 2023. Reasons: compromised peer review; unreliable results or conclusions.

Therefore, scholars tend to use artificial intelligence (AI) approaches to create automatic models to identify AD. AI enables machines to mimic human behaviors. Machine learning (ML) is a subset of AI, which uses statistical methods to enable machines to improve. Deep learning (DL) is a subset of ML. DL makes the computation of deep neural networks feasible. Their relationship is displayed in Figure 1.

**Figure 1:** AI vs. ML vs. DL.

For instance, Plant et al. (2010) used brain region cluster (BRC) as a feature extractor. The authors tested three classifiers and found Bayesian classifier (BC) achieved the best performance. Their average accuracy of BRC-BC reached 92.00%. Savio and Grana (2013) employed the trace of Jacobian matrix (TJM) approach. Their method's average accuracy reached 92.83 ± 0.91% over the Open Access Series of Imaging Studies (OASIS) dataset. Gray et al. (2013) presented a random forest (RF)-based similarity measures for multiple modality classification of AD. The authors included CSF biomarker measures, regional MRI volumes, voxel-based FDG-PET signal intensities, and categorical genetic information. Lahmiri and Boukadoum (2014) used fractal multiscale analysis (FMSA) to extract features. However, their dataset is small, with only 33 images. Zhang (2015) mingled displacement field (DF) with three different support vector machines, and they observed that the twin support vector machine yielded the best performance. Gorji and Haddadnia (2015) combined pseudo-Zernike moment (PZM) with a scaled conjugate gradient (SCG) algorithm. The experimental outcomes showcased that PZM with the order of 30 gave the paramount performance. Li (2018) presented a novel method to combine wavelet entropy (WE) with biogeography-based optimization (BBO). The interclass variance criterion was employed to pick out the single slice from the 3D image. Du (2017) reused PZM for feature extraction. They extracted 256 features from each brain image and substituted SCG with a linear regression classifier (LRC). Sui (2018) presented an eight-layer convolutional neural network (CNN). In traditional CNN, rectified linear unit (ReLU) is the default activation function. The authors replaced ReLU with a new activation function—leaky ReLU (LReLU). They tested three different pooling methods and found that max pooling gave the best performance. Jiang and Chang (2020) further improved the CNN structure and included batch normalization and dropout (BND) technique. Their method is abbreviated as CNN-BND in this paper. Dua et al. (2020) suggested a combination of DL models, which chose some primary models as CNN, recurrent neural networks (RNNs), and long short-term memory (LSTM). Its amalgamation achieved an accuracy of 92.22%. Sutoko et al. (2021) utilized a deep neural network with optimized stepwise feature selection and cross-validation method.

The article "ADVIAN: Alzheimer's Disease VGG-Inspired Attention Network Based on Convolutional Block Attention Module and Multiple Way Data Augmentation" was retracted in 2023. Reasons: compromised peer review; unreliable results or conclusions.

From previous studies, we can observe DL methods can have better performance than traditional ML methods. As mentioned before, DL is a subfield of ML (see Figure 1), but DL powers itself by using a human-like artificial deep neural network to learn and make decisions by itself from given data (Saood and Hatem, 2021).

To further improve the performance of DL, there are three possible ways: (i) depth, (ii) width, and (iii) cardinality of the deep neural networks. We try to improve the performance from the fourth way—the attention mechanism. In all, we propose a novel DL model termed Alzheimer's Disease VGG-Inspired Attention Network (ADVIAN). The contributions of our paper are listed as following four points:

1. A VGG-inspired network (VIN) is particularly designed as the backbone model to identify AD.
2. Convolutional block attention modules are integrated to introduce attention to the VIN.
3. Multiple-way data augmentation is introduced to make test performance more reliable.
4. The test results prove our ADVIAN model is better than 11 state-of-the-art methods.

## Subjects

The dataset we used is already reported in the work of Sui (2018), where 28 AD patients and 98 healthy control (HC) subjects were selected from the OASIS-1 dataset (Ardekani et al., 2013). The selection criterion is to remove individuals under 60 and incomplete observations. Meanwhile, 70 AD subjects were enrolled from local hospitals. Hence, we have a balanced dataset, of which the demographics are itemized in Table 1, where SES means Socioeconomic Status, MMSE Mini-Mental State Exam, and CDR Clinical Dementia Rating.

**Table 1:** Demographics of dataset in this study.

**Trait**	**OASIS**		**Local hospitals**
	**AD (28)**	**HC (98)**	**AD (70)**
Gender (M/F)	9/19	26/72	24/46
Age	77.75 ± 6.99	75.91 ± 8.98	76.34 ± 7.81
SES	2.87 ± 1.29	2.51 ± 1.09	2.89 ± 1.16
Education	2.57 ± 1.31	3.26 ± 1.31	2.63 ± 1.42
MMSE	21.67 ± 3.75	28.95 ± 1.20	21.12 ± 4.62
CDR	1	0	1

*SES, socioeconomic status; CDR, clinical dementia rating; MMSE, mini-mental state exam*.

The article "ADVIAN: Alzheimer's Disease VGG-Inspired Attention Network Based on Convolutional Block Attention Module and Multiple Way Data Augmentation" was retracted in 2023. Reasons: compromised peer review; unreliable results or conclusions.

There are AD researchers favoring Alzheimer's disease neuroimaging initiative (ADNI) (Abuhmed et al., 2021), and many others use OASIS, which is freely accessible, grants sensible demographics for proof of concept, and generalizes easily for forthcoming longitudinal studies.

## Preprocessing

The same preprocessing procedure (shown in Figure 2) applies to all the images in this dataset. First, 1 ≤ *n* ≤ 4 multiple raw scans of the same structural protocol within a single session of the same person is carried out; we obtain *n* volumetric images as *V*_*R*_(*n*).

**Figure 2:** Pipeline of preprocessing.

Second, motion correction (MC) is performed over all the *n* raw images. The motion-corrected images are symbolized as *V*_*MC*_(*n*).

Third, an average image *V*_*A*_ is obtained by averaging all the *n* motion-corrected images, i.e.,


(1) $$\begin{array}{l} V_{A}=\frac{1}{n}\sum_{i=1}^{n}V_{MC}\left(n\right) \end{array}$$

Fourth, gain field (GF) correction is performed. The GF is intensity variations irrelated to the subject's anatomical information. GF may relate to movement, nearly static fields, radiofrequency turbulence, or additional nonsubject causes (Hou, 2006). The image is now symbolized as *V*_*G*_.

Fifth, atlas registration will spatially normalize the image *V*_*G*_ to Talairach atlas (Saletin et al., 2019) and obtain the image *V*_*T*_.

Sixth, a masked image *V*_*M*_ is obtained by removing all the nonbrain voxels. We do not do gray matter/white matter/CSF segmentation at this stage.

Seventh, a key slice is selected *I*_*K*_ from the masked volumetric image *V*_*M*_. There are three view angles: axial, sagittal, and coronal view angles, as shown in Figure 3. In this study, we chose the 80th axial *I*_*K*_ out of 176 slices. The key slice is considered the original image (OI).

**Figure 3:** Slices with different views. **(A)** Axial view, **(B)** Sagittal view, **(C)** Coronal view.

Eighth, data harmonization is performed *via* histogram stretching (HS) (Luo et al., 2021) to counter intersource variability from the difference between our dataset's two sources. The HS is indispensable to normalize the interscan images by increasing the difference between the maximum intensity value and the minimum one in an image. Mathematically, HS (Luo et al., 2021) altered OI *x* to an different image *y* as:


(2) $$\begin{array}{l} y\left(i,j\right)=\frac{x\left(i,j\right)-x_{min}}{x_{max}-x_{min}} \end{array}$$

where *x*_*min*_ and *x*_*max*_ stand for the minimum and maximum intensity values of OI, respectively.

Traditionally, the minimum and maximum correspond to 0 and 100% of the whole grayscale range. In this study, 5 and 95% are employed to replace 0 and 100%, respectively. The motivation is the pixels with the least (0%) and the greatest (100%) values are more susceptible to noises. Using the 95−5% = 90% interval can make HS more dependable than using the 100% interval. After this step, we get harmonized image *I*_*H*_.

The article "ADVIAN: Alzheimer's Disease VGG-Inspired Attention Network Based on Convolutional Block Attention Module and Multiple Way Data Augmentation" was retracted in 2023. Reasons: compromised peer review; unreliable results or conclusions.

Finally, the image *I*_*H*_ is cropped. The cropped image *I* has the size of [176 × 176]. Two key slices of one AD sample and one HC sample are displayed in Figure 4.

**Figure 4:** Samples of our dataset. **(A)** AD, **(B)** HC.

## Methodology

### Background of VGG-16

Transfer learning (TL) stores knowledge gained while solving one problem and applies it to solve a different but related problem (Santana and Silva, 2021). Most pretrained deep neural networks (PDNNs) are trained on a subset of ImageNet database. Those PDNNs could classify images into 1,000 object categories. Hence, using PDNNs for TL is easier and faster than training networks from scratch.

VGG stands for Visual Geometry Group, an academic group at Oxford University. This team presented two famous networks: VGG-16 (Jahangeer and Rajkumar, 2021) and VGG-19 (Sudha and Ganeshbabu, 2021), which are included as library packages of popular programming languages such as Python and MATLAB. This study chooses VGG-16 because it is easier to implement and has less layers, while VGG-16 has similar performance of VGG-19.

Figure 5A displays the structure of VGG-16, which is composed of five conv blocks and three fully connected layers (FCLs). The input of VGG-16 is 224 × 224 × 3. After the 1st convolution block (CB), the output is 112 × 112 × 64. Components of 1st CB are shown in Table 2. The 1st CB can be written as “2 × (64 3 × 3)/2,” which means “2 repetitions of 64 kernels with sizes of 3 × 3 followed by a max pooling with a kernel size of 2 × 2.” Note that (i) ReLU layers are skipped in the following texts as default. (ii) Stride and padding are not included since they can be calculated easily.

**Figure 5:** Structures of three networks. **(A)** VGG-16, **(B)** VIN (Ours), **(C)** ADVIAN (Ours).

**Table 2:** Components of 1st CB “2 × (64 3 × 3) /2” in VGG_16.

**Layer**	**Component**
1	1 convolutional layer with 64 kernels with sizes of 3 × 3 and stride [1, 1] and padding [1, 1, 1, 1]
2	1 ReLU layer
3	1 convolutional layer with 64 kernels with sizes of 3 × 3 and stride [1, 1] and padding [1, 1, 1, 1]
4	1 ReLU layer
5	1 max pooling layer with a kernel size of 2 × 2

The 2nd CB “2 × (128 3 × 3) / 2,” 3rd CB “3 × (256 3 × 3) / 2,” 4th CB “3 × (512 3 × 3) / 2,” and 5th CB “3 × (512 3 × 3) / 2” produce the feature maps (FMs) with sizes of 56 × 56 × 128, 28 × 28 × 256, 14 × 14 × 512, and 7 × 7 × 512, respectively. Afterward, FM is compressed into a column vector of 25,088 neurons and sent into three FCLs with 4,096, 4,096, and 1,000 neurons, respectively.

The article "ADVIAN: Alzheimer's Disease VGG-Inspired Attention Network Based on Convolutional Block Attention Module and Multiple Way Data Augmentation" was retracted in 2023. Reasons: compromised peer review; unreliable results or conclusions.

### VGG-Inspired Network

A VIN is designed, shown in Figure 5B, as our task's backbone network. The VIN is inspired by VGG-16. The VIN contains four CBs and three FCLs. The first CB “2 × [3 × 3, 32] / 2” contains two repetitions of 32 kernels with sizes of 3 × 3 followed by a max pooling with a kernel size of 2 × 2. After four CBs, the size of FM becomes 11 × 11 × 128. The flattening layer vectorizes the FM into a vector with a size of 1 × 1 × 15,488. After three consecutive FCLs, we output a binary code that represents either AD or HC. The structure of the proposed 13-layer VIN is depicted in Table 3, where NWI represents the number of weighted layers, and CH configuration of hyperparameters.

**Table 3:** Arrangement of our 13-layer VIN.

**Index**	**Tag**	**NWL**	**CH**	**Size of FM**
1	Input	0	0	176 × 176 × 1
2	CB-1	2	2 × [3 × 3, 32] / 2	88 × 88 × 32
3	CB-2	2	2 × [3 × 3, 64] / 2	44 × 44 × 64
4	CB-3	3	3 × [3 × 3, 128] / 2	22 × 22 × 128
5	CB-4	3	3 × [3 × 3, 128] / 2	11 × 11 × 128
6	Flatten	0	0	15,488
7	FCL-1	1	200 × 15,488, 200 × 1	200
8	FCL-2	1	200 × 200, 200 × 1	200
9	FCL-3	1	2 × 200, 2 × 1	2

*NWI, number of weighted layers; CH, configuration of hyperparameters; FM, feature map*.

The similarities between the proposed VIN and VGG-16 are itemized in Table 4. Apart from those six similarity aspects (Fernandes, 2021), there are several differences between the proposed VIN and VGG-16. The input of VGG-16 is 224 × 224 × 3, while the input of VIN is 176 × 176 × 1. The output of VGG-16 is 1,000 neurons corresponding to 1,000 categories to be classified, while the output of VIN is 2 neurons because our task is a binary-coded problem. Also, some structural differences exist between those two networks, which can be observed from Figure 5 and Table 4.

**Table 4:** Similarity facets between proposed VIN and VGG-16.

**Key**	**Similarity facet**
A	Employing small convolution kernels with size of (3 × 3)
B	Employ small max pooling kernel with size of (2 × 2)
C	Each CB contains a few repetitions of conv layers followed by a max pooling layer
D	Fully connected layers are put at the end of the deep network
E	Channel number increase as it goes from input to the last conv layer, later decreases as to output.
F	Size of FMs shortens as it goes from input to output

### Human Visual System and Attention Mechanism

To increase the functioning of the recent deep neural networks, numerous investigations are carried out in terms of either width, or depth, or cardinality. For examples, (i) the network structures reported in recent ResNet (He et al., 2016) and DenseNet (Huang et al., 2017) show that deeper network (over 1,000 weighted layers) will have better performance in general; (ii) GoogleNet demonstrates that width (Szegedy et al., 2015) is another critical factor to improve the implementation; Zagoruyko and Komodakis (2016) present wide residual networks, in which the authors reduce the depth and enlarge the width of residual networks; (iii) Xie et al. (2017) expose a new dimension “cardinality” defined as the size of the set of transformations and proves increasing cardinality is more effective than going wider or going deeper.

The article "ADVIAN: Alzheimer's Disease VGG-Inspired Attention Network Based on Convolutional Block Attention Module and Multiple Way Data Augmentation" was retracted in 2023. Reasons: compromised peer review; unreliable results or conclusions.

“Attention” is the fourth possible way to improve the network's performance. There are many papers using attention to improve their networks. Lee et al. (2021) proposed an attention recurrent neural network to estimate severity. Song et al. (2021) presented a coarse-to-fine dual-view attention network for click-through rate prediction. Arora et al. (2021) offered an attention-based deep network for automated skin lesion segmentation.

In all, attention acts an essential role within the human visual system (HVS) (Choi et al., 2020). Figure 6 displays a simplified instance of HVS, in which image formation is first seized by the lens of the human eye's cornea. Thenceforth, the iris makes use of the photoreceptor sensitivity to control the exposure. Afterward, the information stream is passed to cone and rod cells in the retina. At long last, the neural firing is forwarded to the brain for additional handling.

**Figure 6:** Illustration of a simplified HVS.

Human eyes do not endeavor to sort out the whole scenarios captured at one time. In contrast, human beings take the full practice of partial glimpses and fix on salient features selectively to grab a sounder pictorial structure. Thus, the recent attention networks (Oh et al., 2021) embedding attention mechanism will have the advantages of (a) focusing on those critical and salient features, (b) performing more successful than networks without attention mechanism, and (c) become more reliable to noisy inputs than networks without attention mechanism.

### ADVIAN

Woo et al. (2018) presented a new convolutional block attention module (CBAM), which not only informs the neural network model of the regions to focus but also perfects the representation of interests. In their paper, the core idea of CBAM is to improve the 3D FMs by being trained with channel attention and spatial attention, respectively.

CBAM is composed of two consecutive submodules: (i) channel attention module (CAM) and (ii) spatial attention module (SAM). The complete relation between CBAM and its two submodules is exposed in Figure 7.

The article "ADVIAN: Alzheimer's Disease VGG-Inspired Attention Network Based on Convolutional Block Attention Module and Multiple Way Data Augmentation" was retracted in 2023. Reasons: compromised peer review; unreliable results or conclusions.

**Figure 7:** Relation of CBAM and its two submodules.

Suppose we have a provisional input FM of **F** ∈ ℝ^*C* × *H* × *W*^. The CBAM applies 1D CAM ${\text{N}}_{\text{CAM}}\in {\mathbb{R}}^{C\times 1\times 1}$ and a 2D SAM ${\text{N}}_{\text{SAM}}\in {\mathbb{R}}^{1\times H\times W}$ in sequence to the input **F**, as illustrated in Figure 7. Thus, the channel-refined FM and the final FM are obtained as:


(3) $$\begin{array}{l} \{\begin{array}{c} \text{Q}={\text{N}}_{\text{CAM}}\left(\text{P}\right)⊗\text{P}\\ \text{R}={\text{N}}_{\text{SAM}}\left(\text{Q}\right)⊗\text{Q} \end{array} \end{array}$$

where ⊗ means the element-wise multiplication.

If the two operands are not with the same dimension, then the values are transmitted (copied) in such tactics that the spatial attentional values are transmitted by the channel dimension, and the channel attention values are transmitted by the spatial dimension (Fernandes, 2021).

Firstly, CAM is defined. Both max pooling (MP) *f*_*mp*_ and average pooling (AP) *f*_*mp*_ are applied, breeding two features **S**_**ap**_ and **S**_**mp**_.


(4) $$\begin{array}{l} \{\begin{array}{c} {\text{S}}_{\text{a}\text{p}}\;=\;f_{ap}\left(\text{P}\right)\\ {\text{S}}_{\text{m}\text{p}}\;=\;f_{mp}\left(\text{P}\right) \end{array} \end{array}$$

Both are thenceforth sent on to a shared shallow neural network—multilayer perceptron (MLP) (Tiwari, 2021), to produce the output FMs, that are thenceforth united *via* element-wise summation ⊕. Normally, MLP consists of three layers of nodes: an input layer, a hidden layer, and an output layer, as shown in Figure 8A. The united sum is then sent to the sigmoid function β. Precisely,


(5) $$\begin{array}{l} {\text{N}}_{\text{CAM}}\left(\text{P}\right)=\beta \left\{MLP\left[{\text{S}}_{\text{a}\text{p}}\right]⊕MLP\left[{\text{S}}_{\text{m}\text{p}}\right]\right\} \end{array}$$

To decrease the parameter reserves, the number of hidden neurons of MLP is arranged to ${\mathbb{R}}^{C/e_{r}\times 1\times 1}$, where *e*_*r*_ is identified as the reduction ratio. Let ${\text{W}}_{0}\in {\mathbb{R}}^{C/e_{r}\times C}$ and ${\text{W}}_{1}\in {\mathbb{R}}^{C\times C/e_{r}}$ mean the MLP weights, respectively, Equation (5) is updated as:


(6) $$\begin{array}{l} {\text{N}}_{\text{CAM}}\left(\text{P}\right)=\beta \left\{{\text{W}}_{1}\left[{\text{W}}_{0}\left({\text{S}}_{\text{a}\text{p}}\right)\right]⊕{\text{W}}_{1}\left[{\text{W}}_{0}\left({\text{S}}_{\text{m}\text{p}}\right)\right]\right\} \end{array}$$

See **W**_**0**_ and **W**_**1**_ are shared by both **S**_**ap**_ and **S**_**mp**_. Figure 8A shows the flowchart of CAM.

**Figure 8:** Diagram of two submodules in CBAM. **(A)** CAM, **(B)** SAM.

The article "ADVIAN: Alzheimer's Disease VGG-Inspired Attention Network Based on Convolutional Block Attention Module and Multiple Way Data Augmentation" was retracted in 2023. Reasons: compromised peer review; unreliable results or conclusions.

Second, SAM is defined. The spatial attention module **N**_**SAM**_ is a paired phase to the preceding channel attention module **N**_**CAM**_. The AP operation *f*_*ap*_ and MP operation *f*_*mp*_ are harnessed to the channel-refined FM **Q**, and we gain


(7) $$\begin{array}{l} \{\begin{array}{c} {\text{T}}_{\text{a}\text{p}}\;=\;f_{ap}\left(\text{Q}\right)\\ {\text{T}}_{\text{m}\text{p}}\;=\;f_{mp}\left(\text{Q}\right) \end{array} \end{array}$$

Both **T**_**ap**_ and **T**_**mp**_ are two-dimensional FMs: ${\text{T}}_{\text{a}\text{p}}\in {\mathbb{R}}^{1\times H\times W}\wedge {\text{T}}_{\text{m}\text{p}}\in {\mathbb{R}}^{1\times H\times W}$, which are concatenated jointly along the channel dimension as


(8) $$\begin{array}{l} \text{T}=\;f_{con}^{cha}\left({\text{T}}_{\text{a}\text{p}},{\text{T}}_{\text{m}\text{p}}\right) \end{array}$$

where $f_{con}^{cha}$ stands for the concatenation along channel dimension.

The concatenated FM **T** is thenceforth sent into a typical convolution with a size of 7 × 7 *f*_*conv*_. The resultant FM is sent to the sigmoid function β. Altogether, we find:


(9) $$\begin{array}{l} {\text{N}}_{\text{SAM}}\left(\text{Q}\right)=\beta \left\{f_{conv}\left[\text{T}\right]\right\} \end{array}$$

The yielded **N**_**SAM**_(**Q**) is subsequently element-wisely multiplied with **Q**, as displayed in Equation (3). Figure 8B portrays the diagram of SAM.

The previously introduced CBAM is integrated into the proposed VIN network, which renders the proposed ADVIAN shown in Figure 5C, which has the same FM structure as VIN in Figure 5B. The difference between ADVIAN and VIN is that we add CBAM after each CB, and thus we called each block as “conv attention block (CAB),” as shown in Figure 9.

**Figure 9:** Relationship among CAB, CBAM, and CB.

For any FM *P* of each previous CB, the two uninterrupted attention modules (channel and spatial) are attached, coupled with the refined FM *R* which is driven to the succeeding block. Now CAB is made up of one CB and succeeding CBAM module. Comparing Figures 7, 9, we can observe the relationship among CAB, CBAM, and CB.

As default, the softmax function $f_{s}:{\mathbb{R}}^{K}\mapsto {\mathbb{R}}^{K}$ is appended at the end of our model. Suppose the input to the softmax is $z=\left(z_{1},\ldots z_{i},\ldots ,z_{K}\right)\in {\mathbb{R}}^{K}$, we have


(10) $$\begin{array}{l} f_{s}{\left(z\right)}_{i}=\frac{\exp\left(z_{i}\right)}{\sum_{j=1}^{K}exp\left(z_{j}\right)} \end{array}$$

The softmax function can be regarded as the output unit activation function. For classification-oriented deep neural networks, a softmax layer and a classification layer must follow the last FCL. Also, batch normalization (Vrzal et al., 2021) layers are embedded as assisting layers.

The article "ADVIAN: Alzheimer's Disease VGG-Inspired Attention Network Based on Convolutional Block Attention Module and Multiple Way Data Augmentation" was retracted in 2023. Reasons: compromised peer review; unreliable results or conclusions.

### Cross-Validation

Cross-validation (CV) (Albashish et al., 2021) is a resampling route to evaluate AI models on a limited-size dataset. Figure 10 shows the diagram of the *K*-fold CV. The whole dataset is split into *K* folds evenly. Then for *k*th (*k* = 1, …, *K*) trial, the *k*th fold is used for test, and all the other folds (1, …, *k* − 1, *k* + 1, …, *K*) for training. We repeat *K* trials to facilitate each fold used for test only once. The above *K*-fold cross-validation will repeat *R* times. In this study, we set *K* = *R* = 10.

**Figure 10:** Illustration of *K*-fold CV.

### Multiple-Way Data Augmentation

Overfitting may occur due to the small-size dataset in this study. To avoid this, multiple-way data augmentation (MDA) is employed. MDA is a variant of the traditional data augmentation (DA) method. Cheng (Cheng, 2021) presented a 16-way DA to identify COVID-19 chest CT image. In their method, the number of DA is set to *J*_1_ = 8, i.e., eightway different DA were applied to original raw image *r*(*x*) and the horizontally mirrored version *r*^*h*^(*x*).

In this method, we propose an 18-way DA, of which the diagram is displayed in Figure 11. The difference of our 18-way DA against 16-way DA (Cheng, 2021) is that we add the speckle noise (SN) to both *r*(*x*) and *r*^*h*^(*x*), respectively. the SN altered image is defined as


(11) $$\begin{array}{l} r^{SN}\left(x\right)=r\left(x\right)+N_{R}^{*}r\left(x\right), \end{array}$$

where *N*_*R*_ is uniformly distributed random noise. In this study, we set the mean and variance of *N*_*R*_ to 0 and 0.05, respectively.

**Figure 11:** Diagram of 18-way DA.

First, *J*_1_-different DA methods as displayed in Figure 11 are applied to raw training image *r*(*x*). Let **H**_*j*_, *j* = 1, …, *J*_1_ denotes each DA operation, we have the augmented images of raw image *r*(*x*) as


(12) $$\begin{array}{l} {\text{H}}_{j}\left[r\left(x\right)\right],j=1,\ldots ,J_{1} \end{array}$$

Suppose *J*_2_ means the size of generated new images for each DA method, then,


(13) $$\begin{array}{l} |{\text{H}}_{j}\left[r\left(x\right)\right]|=J_{2} \end{array}$$

where || represents the number of elements in the set.

Second, horizontally mirrored image *r*^*h*^(*x*) is generated by


(14) $$\begin{array}{l} r^{h}\left(x\right)=f_{HM}\left[r\left(x\right)\right] \end{array}$$

where *f*_*HM*_ stands for horizontal mirror function.

Third, all the *J*_1_ different DA methods are performed on the mirror image *r*^*h*^(*x*) and generate *J*_1_ different datasets.


(15) $$\begin{array}{l} \{\begin{array}{c} {\text{H}}_{j}\left[r^{h}\left(x\right)\right],j=1,\cdots \;,J_{1}\\ |{\text{H}}_{j}\left[r^{h}\left(x\right)\right]|=J_{2},j=1,\ldots ,J_{1} \end{array} \end{array}$$

Fourth, the raw image *r*(*x*), the horizontally mirrored image *r*^*h*^(*x*), *J*_1_-way datasets of raw image **H**_*j*_[*r*(*x*)], and *J*_1_-way datasets of horizontally mirrored image ${\text{H}}_{j}\left[r^{h}\left(x\right)\right]$ are combined. The final generated dataset from *r*(*x*) is defined as **R**(*x*):


(16) $$\begin{array}{l} r\left(x\right)\mapsto R\left(x\right)=f_{fuse}\left\{\begin{array}{cc} \underset{\begin{array}{l} J_{2}\\ ... \end{array}}{\underset{︸}{\overset{r(x)}{H_{1}[r(x)]}}} & \underset{\begin{array}{l} J_{2}\\ ... \end{array}}{\underset{︸}{\overset{r^{h}(x)}{H_{1}[r^{h}(x)]}}}\\ \underset{J_{2}}{\underset{︸}{H_{J1}[r(x)]}} & \underset{J_{2}}{\underset{︸}{H_{J1}[r^{h}(x)]}} \end{array}\right\} \end{array}$$

where *f*_*fuse*_ is the concatenation function.

The article "ADVIAN: Alzheimer's Disease VGG-Inspired Attention Network Based on Convolutional Block Attention Module and Multiple Way Data Augmentation" was retracted in 2023. Reasons: compromised peer review; unreliable results or conclusions.

Suppose augmentation factor is *J*_3_, which represents the number of images in **R**(*x*), we get


(17) $$\begin{array}{l} J_{3}=\frac{\left|\text{R}\left(x\right)\right|}{\left|r\left(x\right)\right|}=\frac{\left(1+J_{1}\times J_{2}\right)\times 2}{1}=2\times J_{1}\times J_{2}+2 \end{array}$$

**Algorithm 1** recaps the pseudocode of the 18-way DA method. We set *J*_1_ = 9, *J*_2_ = 30; thus, *J*_3_ = 542.

**Algorithm 1:** Pseudocode of 18-way data augmentation.

*Input*	*Import raw preprocessed training image *r*(*x*)*.
*Step A*	*J_1_ geometric/photometric/noise-injection DA transforms* **H**_*j*_ *are utilized on *r*(*x*). We obtain datasets* **H**_*j*_[*r*(*x*)], *j* = 1, …, *J*_1_. *See Eq. (12). Each enhanced dataset comprises *J*_2_ new images. See Eq. (13)*.
*Step B*	*Horizontally mirrored image is obtained by* $r^{h}\left(x\right)=f_{HM}\left[r\left(x\right)\right]$. *See Eq. (14)*.
*Step C*	*J_1_-way DA transforms are implemented on *r*^*h*^(*x*), we obtain datasets* ${\text{H}}_{j}\left[r^{h}\left(x\right)\right],j=1,\cdots \;,J_{1}$. *See Eq. (15)*.
*Step D*	*r(*x*), *r*^*h*^(*x*)*, **H**_*j*_[*r*(*x*)], *j* = 1, …, *J*_1_, *and* ${\text{H}}_{j}\left[r^{h}\left(x\right)\right],j=1,\ldots ,J_{1}$ *are combined. See Eq. (16)*.
*Output*	*Output a new dataset* **R**(*x*). *Its image number is* *J*_3_ = 2 × *J*_1_ × *J*_2_ + 2. *See Eq. (17)*.

### Evaluation

The evaluation was reported on the *R* runs of *K*-fold CV of our 98–98 image dataset. Suppose the image number of each class is *T*_*k*_(*k* = 1, 2). The perfect confusion matrix (CM) is


(18) $$\begin{array}{l} O^{ideal}=\left\{o^{ideal}\right\}=R\times \left[\begin{array}{cc} T_{1} & 0\\ 0 & T_{2} \end{array}\right], \end{array}$$

where the off-diagonal entries of ideal *O*^*ideal*^ are all 0 s, viz., *o*^*ideal*^(*i, j*) = 0, ∀*i* ≠ *j*. The realistic confusion matrix is


(19) $$\begin{array}{l} O=\left\{o\right\}=\left[\begin{array}{cc} o\left(1,1\right) & o\left(1,2\right)\\ o\left(2,1\right) & o\left(2,2\right) \end{array}\right]. \end{array}$$

Now, we define positive (P) and negative (N) classes. The meaning of TP, TN, FP, and FN are shown in Table 5.

The article "ADVIAN: Alzheimer's Disease VGG-Inspired Attention Network Based on Convolutional Block Attention Module and Multiple Way Data Augmentation" was retracted in 2023. Reasons: compromised peer review; unreliable results or conclusions.

**Table 5:** Meanings in measures.

**Abbreviation**	**Full form**	**Symbol**	**Meaning**
P	Positive		AD
N	Negative		HC
TP	True positive	*o*(1, 1)	AD images are classified correctly.
FP	False positive	*o*(2, 1)	HC images are wrongly classified as AD.
TN	True negative	*o*(2, 2)	HC images are classified correctly.
FN	False negative	*o*(1, 2)	AD images are wrongly classified as HC.

Nine measures are used: sensitivity, specificity, precision, accuracy, F1 score, Matthews correlation coefficient (MCC) (Daines et al., 2020), Fowlkes–Mallows index (FMI) (Monteiro et al., 2018), receiver operating characteristic (ROC), and area under the curve (AUC). The first four measures are defined as


(20) $$\begin{array}{l} \{\begin{array}{cc} \text{Sen}=\frac{o\left(1,1\right)}{o\left(1,1\right)+o\left(1,2\right)} & \text{Spc}=\frac{o\left(2,2\right)}{o\left(2,2\right)+o\left(2,1\right)}\\ \text{Prc}=\frac{o\left(1,1\right)}{o\left(1,1\right)+o\left(2,1\right)} & \text{Acc}=\frac{o\left(1,1\right)+o\left(2,2\right)}{o\left(1,1\right)+o\left(2,2\right)+o\left(1,2\right)+o\left(2,1\right)} \end{array} \end{array}$$

and the middle three measures are defined as:


(21) $$\begin{array}{l} F_{1}=2\times \frac{\text{Sen}\times \text{Prc}}{\text{Sen}+\text{Prc}}=\frac{2\times o\left(1,1\right)}{2\times o\left(1,1\right)+o\left(1,2\right)+o\left(2,1\right)} \end{array}$$

(22) $$\begin{array}{l} \text{MCC}=\frac{o\left(1,1\right)\times o\left(2,2\right)-o\left(2,1\right)\times o\left(1,2\right)}{\sqrt{\left[o\left(1,1\right)+o\left(2,1\right)\right]\times \left[o\left(1,1\right)+o\left(1,2\right)\right]\times \left[o\left(2,2\right)+o\left(2,1\right)\right]\times \left[o\left(2,2\right)+o\left(1,2\right)\right]}} \end{array}$$

(23) $$\begin{array}{l} \text{FMI}=\sqrt{\text{Sen}\times \text{Prc}}=\sqrt{\frac{o\left(1,1\right)}{o\left(1,1\right)+o\left(1,2\right)}\times \frac{o\left(1,1\right)}{o\left(1,1\right)+o\left(2,1\right)}} \end{array}$$

The above measures are calculated in the mean and standard deviation (MSD) format. Besides, ROC is a curve to measure a binary classifier with varying discrimination thresholds. The ROC curve is created by plotting the sensitivity against 1-specificity. The AUC is calculated based on the ROC curve.

The article "ADVIAN: Alzheimer's Disease VGG-Inspired Attention Network Based on Convolutional Block Attention Module and Multiple Way Data Augmentation" was retracted in 2023. Reasons: compromised peer review; unreliable results or conclusions.

## Experiments and Results

### Multiple-Way Data Augmentation

Figure 12 displays the part of 18-way DA results (i.e., **H**_*j*_[*r*(*x*)], *j* = 1, …, *J*_1_) if we take Figure 4A as the raw image *r*(*x*). From Figure 12, we can observe that this 18-way DA improves the diversity of our training set, which will make our classifier model more robust. In the following experiments, we shall prove this robustness.

**Figure 12:** Results of data augmentation. **(A)** Horizontal shear, **(B)** Vertical shear, **(C)** Image rotation, **(D)** Gamma correction, **(E)** Random translation, **(F)** Scaling, **(G)** Gaussian noise, **(H)** Salt-and-pepper noise, **(I)** Speckle noise.

### Statistical Analysis

The results of 10 runs of 10-fold cross-validation of our model ADVIAN are itemized in Table 6. The sensitivity and specificity reach 97.65 ± 1.36 and 97.86 ± 1.55, respectively. Its precision and accuracy are 97.87 ± 1.53 and 97.76 ± 1.13, respectively. The F1 score, MCC, and FMI are obtained as 97.75 ± 1.13, 95.53 ± 2.27, and 97.76 ± 1.13, respectively. We can see that all the seven indicators of our model are above 95%. The ROC curve is displayed in Figure 14B, and the AUC is 0.9852.

**Table 6:** Results of proposed ADVIAN model.

**Run**	**Sen**	**Spc**	**Prc**	**Acc**	**F1**	**MCC**	**FMI**
1	100.00	97.96	98.00	98.98	98.99	97.98	98.99
2	97.96	96.94	96.97	97.45	97.46	94.90	97.46
3	97.96	95.92	96.00	96.94	96.97	93.90	96.97
4	97.96	100.00	100.00	98.98	98.97	97.98	98.97
5	95.92	98.98	98.95	97.45	97.41	94.94	97.42
6	97.96	95.92	96.00	96.94	96.97	93.90	96.97
7	97.96	98.98	98.97	98.47	98.46	96.94	98.46
8	95.92	96.94	96.91	96.43	96.41	92.86	96.41
9	95.92	96.94	96.91	96.43	96.41	92.86	96.41
10	98.98	100.00	100.00	99.49	99.49	98.98	99.49
MSD	97.65 ± 1.36	97.86 ± 1.55	97.87 ± 1.53	97.76 ± 1.13	97.75 ± 1.13	95.53 ± 2.27	97.76 ± 1.13

### Effect of 18-Way DA

To validate the importance of 18-way DA, we carry out an ablation study in which we remove 18-way DA from our model and observe the performance change. After another 10 runs of 10-fold CV, the performances decrease to a sensitivity of 92.45 ± 2.21, a specificity of 94.18 ± 1.99, a precision of 94.13 ± 1.81, an accuracy of 93.32 ± 1.16, and an F1 score of 93.25 ± 1.20. The MCC and FMI decrease to 86.69 ± 2.31 and 93.27 ± 1.20, respectively. The result of comparison with and without 18-way DA is shown in Figure 13. The ROC curve comparison is shown in Figure 14, where we can observe that AUC without 18-way DA is only 0.9603 (Figure 14A) and AUC with 18-way DA is 0.9852 (Figure 14B).

**Figure 13:** Error bar of the effectiveness of 18-way DA (w/ means with wo/ means without).

**Figure 14:** ROC curves of the effectiveness of 18-way DA (w/ means with wo/ means without). **(A)** wo/MDA, **(B)** w/MDA.

The article "ADVIAN: Alzheimer's Disease VGG-Inspired Attention Network Based on Convolutional Block Attention Module and Multiple Way Data Augmentation" was retracted in 2023. Reasons: compromised peer review; unreliable results or conclusions.

### Method Comparison

To further show the proposed ADVIAN model's effectiveness, we compare it with 11 existing algorithms on the same dataset by 10 runs of 10-fold CV. The comparison methods include BRC-BC (Plant et al., 2010), TJM (Savio and Grana, 2013), RF (Gray et al., 2013), FMSA (Lahmiri and Boukadoum, 2014), DF (Zhang, 2015), PZM-SCG (Gorji and Haddadnia, 2015), BBO (Li, 2018), PZM-LRC (Du, 2017), CNN-LReLU (Sui, 2018), CNN-BND (Jiang and Chang, 2020), and CNN-RNN-LSTM (Dua et al., 2020). The comparison is displayed in Table 7, with the bar plot shown in Figure 15.

**Table 7:** Comparison with other methods.

**Algorithm**	**Sen**	**Spc**	**Prc**	**Acc**	**F1**	**MCC**	**FMI**
BRC-BC (Plant et al., 2010)	92.96 ± 1.63	88.78 ± 1.86	89.25 ± 1.59	90.87 ± 1.11	91.05 ± 1.09	81.83 ± 2.22	91.08 ± 1.09
TJM (Savio and Grana, 2013)	88.27 ± 3.27	92.45 ± 2.37	92.20 ± 2.03	90.36 ± 1.31	90.13 ± 1.44	80.88 ± 2.53	90.18 ± 1.41
RF (Gray et al., 2013)	87.86 ± 2.18	88.67 ± 1.70	88.60 ± 1.55	88.27 ± 1.36	88.21 ± 1.41	76.56 ± 2.72	88.22 ± 1.41
FMSA (Lahmiri and Boukadoum, 2014)	90.31 ± 2.32	87.86 ± 2.47	88.21 ± 1.93	89.08 ± 1.08	89.21 ± 1.08	78.25 ± 2.13	89.23 ± 1.07
DF (Zhang, 2015)	90.61 ± 1.65	93.16 ± 1.18	93.00 ± 1.08	91.89 ± 0.70	91.78 ± 0.75	83.83 ± 1.39	91.79 ± 0.74
PZM-SCG (Gorji and Haddadnia, 2015)	92.96 ± 1.63	92.65 ± 1.79	92.72 ± 1.57	92.81 ± 0.70	92.82 ± 0.69	85.65 ± 1.40	92.83 ± 0.69
BBO (Li, 2018)	91.73 ± 1.83	91.43 ± 2.21	91.52 ± 1.89	91.58 ± 0.60	91.60 ± 0.56	83.22 ± 1.21	91.61 ± 0.57
PZM-LRC (Du, 2017)	93.37 ± 1.82	92.76 ± 2.01	92.83 ± 1.81	93.06 ± 1.30	93.08 ± 1.29	86.15 ± 2.59	93.09 ± 1.29
CNN-LReLU (Sui, 2018)	97.35 ± 1.88	96.94 ± 1.08	96.97 ± 1.01	97.14 ± 0.87	97.14 ± 0.90	94.31 ± 1.72	97.15 ± 0.89
CNN-BND (Jiang and Chang, 2020)	97.04 ± 1.55	97.35 ± 1.29	97.36 ± 1.24	97.19 ± 0.88	97.19 ± 0.89	94.41 ± 1.73	97.19 ± 0.88
CNN-RNN-LSTM (Dua et al., 2020)	92.65 ± 1.65	92.35 ± 1.30	92.38 ± 1.19	92.50 ± 1.02	92.51 ± 1.04	85.02 ± 2.04	92.51 ± 1.04
Ours	97.65 ± 1.36	97.86 ± 1.55	97.87 ± 1.53	97.76 ± 1.13	97.75 ± 1.13	95.53 ± 2.27	97.76 ± 1.13

**Figure 15:** Bar plot of all methods.

In Figure 15, we move the MCC to the leftmost since its value range is smaller than the other six measures. We sort all algorithms in terms of MCC, and the sorted list can be observed at the bottom left corner of Figure 15. The 3D bar plot clearly shows that our method achieves better results than all 11 state-of-the-art methods.

This paper is mainly focusing on methodological improvements. We shall try to combine DL with individual anatomical brain regions [such as medial temporal lobe (Chen et al., 2016a), etc.] and brain network connectively patterns (Chen et al., 2016b) in AD patients.

The article "ADVIAN: Alzheimer's Disease VGG-Inspired Attention Network Based on Convolutional Block Attention Module and Multiple Way Data Augmentation" was retracted in 2023. Reasons: compromised peer review; unreliable results or conclusions.

## Conclusions

This paper proposes a novel VGG-inspired network as the mainstay and combines the attention mechanism with VIN to produce a new ADVIAN deep-learning model to detect AD. The 18-way DA is harnessed to prevent overfitting in the training set. The experiments revealed the usefulness and superiority of this proposed ADVIAN method.

Nevertheless, there are several shortcomings. First, this model did not go through strict clinical environment tests. Second, the dataset is relatively small. Third, the AI output is hard to understand for human experts.

Correspondingly, we may carry out the following researches in the future. We shall deploy our ADVIAN to hospitals to receive feedback directly from clinical doctors. Meanwhile, we will try to collect more AD data. Finally, explainable AI will be included in our future studies.

## Data Availability Statement

The original contributions presented in the study are included in the article/supplementary material, further inquiries can be directed to the corresponding authors.

## Author Contributions

S-HW: conceptualization, methodology, software, data curation, writing (original draft), and funding acquisition. QZ: writing (original draft), writing (review and editing), and visualization. MY: resources, writing (review and editing), supervision, project administration, and funding acquisition. Y-DZ: methodology, software, formal analysis, validation, resources, writing (original draft), writing (review and editing), supervision, project administration, and funding acquisition. All authors contributed to the article and approved the submitted version.

## Conflict of Interest

The authors declare that the research was conducted in the absence of any commercial or financial relationships that could be construed as a potential conflict of interest.

## Abbreviations

AD: Alzheimer's disease
ADNI: Alzheimer's disease neuroimaging initiative
AI: artificial intelligence
AP: average pooling
AUC: area under the curve
CAM: channel attention module
CBAM: convolutional block attention module
CDR: clinical dementia rating
CH: configuration of hyperparameters
CT: computed tomography
CV: cross-validation
DL: deep learning
FCL: fully connected layer
FM: feature map
FMI: Fowlkes–Mallows index
GF: gain field
HS: histogram stretching
HVS: human visual system
MC: motion correction
MCC: matthews correlation coefficient
ML: machine learning
MLP: multilayer perceptron
MMSE: mini-mental state exam
MP: max pooling
MRI: magnetic resonance imaging
MSD: mean and standard deviation
NWL: number of weighted layers
OASIS: open access series of imaging studies
OI: original image
PDNN: pretrained deep neural network
PET: positron emission tomography
ReLU: rectified linear unit
ROC: receiver operating characteristic
SAM: spatial attention module
SES: socioeconomic status
SN: speckle noise
TL: transfer learning
VGG: visual geometry group.
